The article "Occlusion with Bronchial Covered Stent in the Management of Bronchial Stump Fistula after Right Middle and Lower Lobectomy: A Case Report and Literature Review" was published in 2021. Journal: Zhongguo Fei Ai Za Zhi.

# 支气管覆膜支架封堵治疗右肺中下叶切除术后支气管残端瘘经验1例

**DOI:** 10.3779/j.issn.1009-3419.2021.101.11

**Published:** 2021-04-20

**Authors:** 淼 黄, 方亮 鲁, 少雷 李, 宇权 裴, 亮 王, 跃 杨

**Affiliations:** 100142 北京，北京肿瘤医院胸外二科 Department of Thoracic Surgery II, Peking University Cancer Hospital, Beijing 100142, China

**Keywords:** 右肺中下叶切除术, 支气管残端瘘, 覆膜支架, Right middle and lower lobectomy, Bronchial stump fistula, Covered stent

## Abstract

**背景与目的:**

支气管胸膜瘘是临床上较为严重且罕见的术后并发症之一，尤其是肺叶/全肺切除术后支气管残端瘘，处理起来较为棘手。常见治疗方案包括内科保守治疗联合外科手术，但由于瘘口迁延不愈导致胸腔持续与外界相通，患者容易合并严重的胸腔感染及呼吸衰竭等合并症，以至于身体状况无法耐受二次手术。而内镜下治疗，为该合并症的治疗提供了新的思路。

**方法:**

回顾性分析了北京大学肿瘤医院胸外二科2016年6月收治的1例右肺鳞癌患者的诊断、治疗过程，并文献复习。

**结果:**

患者男性，65岁，因“咳嗽伴痰中带血3月余”入院，胸部计算机断层扫描提示右肺下叶软组织密度肿块影，气管镜提示右肺中叶及下叶基底段开口可见肿物，活检病理证实为鳞癌。诊断考虑：右肺中下叶鳞癌(cT2aN2，IIIa期)。患者接受了吉西他滨+顺铂方案新辅助化疗2个周期，评效为疾病稳定(stable disease, SD)。末次化疗结束4周之后，患者接受了胸腔镜辅助右肺中下叶切除、纵隔淋巴结清扫术。术后第5天患者出现急性呼吸窘迫综合征(acute respiratory distress syndrome, ARDS)再次气管插管转入重症加强护理病房(intensive care unit, ICU)，并给予激素冲击治疗。术后第7天患者出现右肺中间干支气管残端瘘，但由于合并ARDS，患者身体情况无法耐受二次手术。遂于体外人工膜肺(extracorporeal membrane oxygenation, ECMO)支持下，经硬质支气管镜在中间干支气管残端置入一枚定制的覆膜、可膨胀金属铰链支架，并成功封堵。由于患者的ARDS未见好转，出现不可逆的肺间质纤维化，经过系统的抗感染治疗之后，患者成功接受了双肺移植手术。

**结论:**

内镜下放置覆膜支架是一种简单、安全、有效的支气管残端瘘闭合术。当患者的临床情况不适合立即手术时，内镜下支架植入可作为一种优选的治疗方法，为后续治疗创造机会。

## Abstract (en)

**Background and objective:**

Bronchopleural fistula (BPF) is one of the most serious and rare postoperative complications, especially the bronchial stump fistula after lobectomy/pneumonectomy. Common treatment options include conservative medical treatment combined with surgery. However, due to the delayed healing of the fistula, the chest cavity continues to communicate with the outside world, and the patient is prone to complicated with severe thoracic infection and respiratory failure, so that the physical condition can hardly tolerate the second surgical procedure. Endoscopic treatment provides a new option for the treatment of this complication.

**Methods:**

A case of right pulmonary squamous cell carcinoma was admitted to the Department of Thoracic Surgery II, Peking University Cancer Hospital in June 2016. The diagnosis and treatment was retrospectively analyzed, and the literature was reviewed.

**Results:**

A 65 year old male patient was admitted to hospital because of "cough with blood in sputum for 3 months". Chest computed tomography (CT) showed soft tissue density mass shadow in the right lower lobe. A tumor could be seen in the opening of the right middle lobe and basal segment of lower lobe. Biopsy confirmed squamous cell carcinoma. Diagnosis consideration: squamous cell carcinoma of the middle and lower lobe of the right lung (cT2aN2, IIIa). Patients received gemcitabine plus cisplatin neoadjuvant chemotherapy for 2 cycles, and the effect of chemotherapy showed stable disease (SD). Four weeks after chemotherapy, the patient underwent video-assisted thoracic surgery (VATS) assisted right middle and lower lobectomy and mediastinal lymph node dissection. On the 5^th^ day after operation, the patient developed acute respiratory distress syndrome (ARDS) and was transferred to intensive care unit (ICU) again after endotracheal intubation. On the 7^th^ day after operation, the patient developed a right intermediate trunk bronchial stump fistula, but due to ARDS, the patient's physical condition could not tolerate the second operation. Under the support of extracorporeal membrane oxygenation (ECMO), a membrane covered, expandable, hinged stent was inserted into the intermediate trunk bronchial stump through rigid bronchoscope, and was successfully blocked. Due to no improvement in ARDS and irreversible pulmonary interstitial fibrosis, the patient received double lung transplantation successfully after systemic anti-infection treatment.

The article "Occlusion with Bronchial Covered Stent in the Management of Bronchial Stump Fistula after Right Middle and Lower Lobectomy: A Case Report and Literature Review" was published in 2021. Journal: Zhongguo Fei Ai Za Zhi.

**Conclusion:**

Endoscopic implantation of covered stent is a simple, safe and effective method for closure of bronchial stump fistula. When the patient's clinical situation is not suitable for immediate surgery, endoscopic stent implantation can be used as a preferred treatment method to create opportunities for follow-up treatment.

## 1 病例资料

患者男性，65岁，主因“间断咳嗽伴痰中带血3月余”，于2016年4月就诊于我院。2016年1月起患者无诱因出现间断咳嗽，干咳为主，伴少量黄痰，偶尔出现痰中带血丝，咳嗽无明显时相性特点，无胸痛、发热、呼吸困难等不适。后就诊于当地医院，行胸部计算机断层扫描(computed tomography, CT)检查发现右肺占位性病变，怀疑恶性。于当地医院完善纤维支气管镜检查，于右肺中叶及下叶基底段支气管开口可见肿物，活检病理提示：鳞癌。为进一步诊治来我院就诊，完善全身正电子发射型计算机断层显像(positron emission tomography, PET)-CT提示：右下肺门区可见一高代谢肿块(图 1A)，大小约3.4 cm×3.4 cm，最大标准化摄取值(maximal standard uptake value, SUVmax)9.1，纵隔内见多个淋巴结影，较大者约1.1 cm×0.8 cm，未见异常放射性浓聚; 全身其他部位未见异常浓聚灶。气管镜活检组织切片送我院病理科会诊报告显示：(右中下叶)低分化鳞状细胞癌。患者既往患有2型糖尿病5年余，口服二甲双胍及阿卡波糖，血糖控制满意; 患高血压5年，口服波依定及比索洛尔，血压控制良好; 吸烟50年，平均40支/天，已戒烟2周。否认药物及食物过敏史。初步诊断为：①右肺中下叶鳞癌(cT2aN2，IIIa期); ②高血压病; ③2型糖尿病; ④左肾上腺结节。

**图 1:** 新辅助化疗前后影像学扫描图像。A：新辅助化疗前PET-CT扫描图像，肿物大小3.4 cm×3.4 cm，SUVmax值9.1; B：新辅助化疗后CT扫描图像，肿物大小3.2 cm×3.1 cm，评效疾病稳定。 The images were scanned before and after neoadjuvant chemotherapy. A: PET-CT scan image before neoadjuvant chemotherapy showed tumor size of 3.4 cm×3.4 cm and SUVmax value of 9.1; B: CT scan image after neoadjuvant chemotherapy showed tumor size of 3.2 cm×3.1 cm and stable disease. PET: positron emission tomography; CT: computed tomography; SUVmax: maximal standard uptake value.

患者于门诊完善心电图、血常规、肝肾功能、凝血等未见明显异常，遂建议患者行术前新辅助化疗，具体方案为吉西他滨(1, 250 mg/m^2^ d1+d8)+顺铂(75 mg d1、d2)。患者于2016年4月12日开始行2周期新辅助化疗，过程较顺利，化疗期间曾出现轻度恶心呕吐，给予对症治疗，未出现脱发、骨髓抑制等不良反应。化疗2个周期后复查胸部CT，肿物大小3.2 cm×3.1 cm，评效为疾病稳定(stable disease, SD)(图 1B)。进一步完善肺功能、心脏超声、颈部及下肢血管超声、24 h动态心电图等检查，提示心肺功能大致正常，未见明确手术禁忌。患者末次化疗结束4周之后再次办理入院，完善术前准备，于2016年6月27日在全麻下行胸腔镜辅助右肺中下叶切除术、纵隔淋巴结清扫术、预防性胸导管结扎术。术中离断血管及支气管所使用的器械均为美国美敦力公司生产的腔镜下吻合器(Endo-GIATM Reloads with Tri-Staple^TM^ Technology)。手术结束之后仔细检查创面未见明显出血，冲洗胸腔，嘱麻醉师双肺通气之后，未见明显漏气，放置24 F引流管行胸腔闭式引流术。手术共耗时3.5 h，术中出血约100 mL。

术后第1日，患者生命体征平稳，胸腔引流880 mL，暗红色血性液。给予苏灵2 U止血治疗，同时静脉补充白蛋白减少渗出，常规给予镇痛、抑酸、预防性抗炎、化痰等药物治疗。术后第2日，引流750 mL，第3日引流450 mL，淡红色血性液，咳嗽时胸瓶未见气泡溢出。术后第3日下午，患者进食鸡汤后，胸腔引流液变为橘红色稍浑浊液体，考虑乳糜漏，嘱严格进食素食。术后第5日，全天胸腔引流量75 mL，形状恢复为淡红色血性液。

术后第5日上午10时左右，患者诉呼吸困难、咳痰无力，视诊患者神志清楚，精神稍差，伴气促。心电监护显示心率102次/分，鼻导管吸氧情况下，脉搏血氧饱和度(pulse oxygen saturation, SpO_2_)88%-90%。听诊双肺呼吸音粗，可闻及湿罗音及哮鸣音。立即给予床旁气管镜吸痰治疗，主气管及左右主支气管开口内可见中等量稀薄样痰液，吸痰后听诊双肺呼吸音稍好转，SpO_2_为85%-90%。急查床旁胸片，可见双肺纹理明显增粗。急查血气分析，动脉血氧分压(arterial oxygen partial pressure, PaO_2_)为53.4 mmHg，动脉血二氧化碳分压(arterial partial pressure of carbon dioxide, PaCO_2_)为40.9 mmHg，诊断为Ⅰ型呼吸衰竭。急诊行肺动脉CT血管造影技术检查，未见肺动脉血栓形成，双肺呈现出弥漫性水肿、渗出表现，诊断考虑为：急性呼吸窘迫综合征(acute respiratory distress syndrome, ARDS)。患者血氧饱和度进行性下降，心率加快120次/分，紧急呼叫麻醉科气管插管后，将患者转入重症加强护理病房(intensive care unit, ICU)，接呼吸机辅助通气，同时给予镇静、降压、平喘、化痰、抑酸、预防性抗凝等药物支持治疗。请呼吸科会诊，诊断考虑为急性肺损伤，建议激素冲击治疗(注射用甲泼尼龙琥珀酸钠120 mg/d，3 d)，并联合应用亚胺培南西司他丁纳+万古霉素抗感染，同时每日行支气管镜下吸痰清除气道分泌物。监测胸片提示患者病情趋于稳定。

术后第7日下午15:00左右，患者出现血氧饱和度下降，胸腔引流瓶中可见大量连续气泡溢出，右侧胸壁皮下气肿，听诊发现右肺呼吸音完全消失，急查床旁胸片：右侧气胸，右肺完全性不张。床旁支气管镜可见右侧中间干支气管残端完全开放状态，考虑合并支气管胸膜瘘——右侧中间干支气管残端瘘，瘘口直径约15 mm。遂行气管切开术，将气管插管插入左主支气管行单肺通气，以保证有效气体交换，并上调呼吸机参数，SpO_2_维持在92%-95%。因患者合并ARDS及肺部感染，身体情况无法耐受二次手术，建议患者家属考虑行内镜下支架封堵治疗，需定制一枚覆膜、可膨胀金属铰链支架(图 2A)。

**图 2:** 经支气管镜下支架置入封堵术。A：定制的覆膜、可膨胀的金属铰链支架; B：硬质支气管镜; C：高频喷射呼吸机; D：支架成功置入支气管瘘口所在位置。 Occlusion with bronchial stent under bronchoscopy. A: A personalized membrane covered, expandable, hinged, metal stent; B: rigid bronchoscope; C: high frequency jet respirometer; D: The stent was successfully placed at the site of the bronchial fistula.

术后第10天，拟在全麻下行“经支气管镜右侧中间干支气管残端瘘口支架置入术”。术中经气管切开处拔出气管插管更换硬质支气管镜(图 2B)，拟在高频喷射呼吸机(图 2C)支持下行内镜下操作时，患者血氧进行性下降，出现心跳骤停，立即行胸外按压，3 min之后患者恢复自主心律。考虑患者无法耐受操作，向家属交代病情后，同意术中放置体外膜肺(extracorporeal membrane oxygenation, ECMO)后，再次尝试行支架置入术。遂经股静脉及颈静脉置管，行VV模式ECMO置入术，接长效膜式氧合器之后，SpO_2_升至100%。再次尝试行硬质支气管镜下支架置入术，操作过程顺利，支架顺利放置在右侧中间干支气管残端(图 2D)，后患者安返ICU病房。

支架术后第2天，患者ECMO支持+呼吸机辅助通气状态，吸入气中的氧浓度分数(fraction of inspired oxygen, FiO_2_)为60%，PaO_2_为82 mmHg，动脉血二氧化碳分压PaCO_2_为39 mmHg，SpO_2_为98%。胸腔引流瓶中气泡明显减少，复查床旁胸片提示：支架位置良好(图 3B)，右肺逐渐复张(图 3C)，考虑支架封堵治疗有效。减停镇静药之后，评估患者意识，患者有睁眼、点头动作，呼之可应。因患者合并严重肺部感染、脓胸，患者出现间断高热，降钙素原进行性升高(最高达19.93 ng/mL)，继续调整抗感染治疗药物，并联合丙种球蛋白治疗之后，体温、血象、降钙素原逐渐将至正常。支架术后25 d，因患者ARDS、双肺间质纤维化未见明显好转迹象，患者家属自行联系转院，后行双肺移植手术治疗。

**图 3:** 支架置入前后患者胸片情况。A：支气管残端瘘发生之后，右全肺不张; B：支架置入术后第1天，胸片上支架所在位置; C：支架封堵残端瘘口之后，右肺逐渐复张。 Chest X-ray before and after stent implantation. A: Right lung atelectasis after the bronchial stump fistula occurred; B: Location of the stent on chest X-ray on the first day after stent implantation; C: The right lung gradually re-expanded after the stent blocked the stump fistula.

The article "Occlusion with Bronchial Covered Stent in the Management of Bronchial Stump Fistula after Right Middle and Lower Lobectomy: A Case Report and Literature Review" was published in 2021. Journal: Zhongguo Fei Ai Za Zhi.

## 2 讨论

近年来，尽管外科手术技术和围手术期管理取得了长足的进步，肺切除术后的并发症发生率仍在25%左右^[1]^。支气管胸膜瘘(bronchopleural fistula, BPF)是肺外科术后致命的并发症之一，既往报道^[2-4]^显示，BPF的发生率为1%-4%，死亡率为16%-72%。BPF常见危险因素，包括：右全肺切除术、术前大剂量放疗、术前合并糖尿病、术前感染等，由于肺叶切除术后BPF较全肺切除术后BPF发生率及围术期死亡率更低，故肺叶切除术后的BPF鲜有报道。据Nagahiro等^[5]^报道，肺叶切除术后BPF的发生率为1.56%，死亡率高达41.7%。高死亡率的主要原因是难治性肺部感染、持续性脓胸、合并ARDS和败血症等。多因素分析显示鳞状细胞癌、术前化疗、下叶或中下叶切除术是肺癌术后BPF的重要危险因素。肺鳞状细胞癌大多为中央型，与周围型肺癌相比，支气管周围需要更广泛的切除，这可能导致支气管残端的有效血流量减少，进而导致BPF。术前化疗可能会影响支气管残端的愈合，因为化疗常导致肺门组织及纵隔纤维化^[6]^，使得术中支气管解剖和保留支气管血供更加困难。下叶或中下叶切除后，由于残端与纵隔软组织的距离更长，支气管残端血流减少可能比上叶切除后更为严重。

多学科综合治疗模式已被证实是IIIa期-IIIb期非小细胞肺癌(non-small cell lung cancer, NSCLC)患者的首选治疗方法。对于部分局部进展期NSCLC患者，术前行新辅助化疗有助于减少肿瘤负荷、增加手术R0切除率并降低术后复发风险^[7, 8]^。尽管有这些积极的作用，化疗药物的毒性对于术后组织愈合仍具有潜在的不利影响，特别是支气管吻合口层面。结合以上分析，本例患者合并有鳞状细胞癌、术前化疗、中下叶切除术、术前合并糖尿病等BPF高危因素，且因为术后出现ARDS需二次气管插管接呼吸机辅助通气，并使用激素冲击治疗，这两项因素亦会增加支气管胸膜瘘发生风险，故该患者的确为BPF高危患者。

在BPF发生之初，若发现及时，且患者一般情况良好，二次手术缝合加固支气管残端是一个较为理想的治疗方法。但BPF的直接后遗症是呼吸功能不全、吸入性肺炎以及脓胸，进而引起严重的败血症，危及生命，无法耐受全麻手术。此种情况之下，内镜下治疗手段更为可取，以避免麻醉和手术的风险。Imai等^[9]^回顾性分析了45例肺叶切除术后支气管胸膜瘘患者，29例(64%)实施了单纯内镜下治疗，9例通过支气管镜下密封胶(如聚乙醇酸纤维蛋白胶等)封堵治疗得以治愈。研究发现，< 3 mm的瘘口对内镜下密封胶治疗反应特别好，但超过8 mm的瘘口不适合行单纯内镜下密封胶治疗，而应考虑内镜下支架置入或联合外科手术治疗。

目前，已经有多种气道支架可供选择，常用的如硅胶管支架(Dumon支架)和可膨胀金属支架，文献报道均有成功治疗BPF的先例^[10]^，但这两种支架均需要在全麻下经硬质支气管镜放置到瘘口所在的位置。覆膜、可膨胀金属铰链支架与硅胶支架相比，其优势在于，金属支架更容易固定，减少移位，从而避免反复支气管镜调整支架位置，而且金属支架强度更大，不易断裂，表面覆膜可以有效封堵瘘口。金属支架内的网状物可以诱导组织增殖和肉芽组织的生长，促进瘘口愈合，然而，这种愈合往往需要2个月甚至更久的时间^[11]^。这种支架的局限性还在于，覆膜支架可能会阻碍支气管黏膜纤毛对分泌物的清除，从而导致痰液潴留，而支架的放置和取出则有可能会损伤气管或声带，并导致出血或气道阻塞等并发症。

本例患者因支气管残端瘘口较大(约15 mm)，因此选用的是覆膜金属支架，且封堵效果良好。因为瘘口较大，支气管镜下支架封堵只是一个临时的过渡性治疗方法，为后续控制肺部感染及脓胸创造了有利条件，帮助患者改善临床状况，为接下来的手术治疗提供了充足的时间和空间。

总之，目前还没有比较不同方案治疗BPF的随机对照研究，加上患者病情的复杂性，几乎所有的相关文献都是个案报道及个人经验总结。因此，临床上对于BPF的处理较为棘手，缺乏较为理想的治疗方案。而内镜下治疗，为BPF的治疗提供了新的思路。本案例报道的意义在于，内镜下放置覆膜支架是一种简单、安全、有效的支气管残端瘘闭合术。当患者的临床情况不适合立即手术时，内镜下支架植入可作为一种优选的治疗方法，为后续治疗创造机会。

## References

[1] Stephan F, Boucheseiche S, Hollande J (2000). Pulmonary complications following lung resection: a comprehensive analysis of incidence and possible risk factors. Chest.

[2] Asamura H, Naruke T, Tsuchiya R (1992). Bronchopleural fistulas associated with lung cancer operations. Univariate and multivariate analysis of risk factors, management, and outcome. J Thorac Cardiovasc Surg.

[3] Vester SR, Faber LP, Kittle CF (1991). Bronchopleural fistula after stapled closure of bronchus. Ann Thorac Surg.

[b4] 4Ponn RB. Complications of pulmonary resection. In: Shields TW, editor. General thoracic surgery. Philadelphia: Lippincott, Willams & Wilkins, 2005: 554-586.

The article "Occlusion with Bronchial Covered Stent in the Management of Bronchial Stump Fistula after Right Middle and Lower Lobectomy: A Case Report and Literature Review" was published in 2021. Journal: Zhongguo Fei Ai Za Zhi.

[5] Nagahiro I, Aoe M, Sano Y (2007). Bronchopleural fistula after lobectomy for lung cancer. Asian Cardiovasc Thorac Ann.

[b6] 6Singhal S, Shrager JB, Kaiser LR. Multimodality therapy for non- small-cell lung cancer. In: Shields TW ed, General Thoracic Surgery. Philadelphia: Lippincott Willams & Wilkins, 2005: 1653-1679.

[7] Martins RG, D'Amico TA, Loo BW Jr (2012). The management of patients with stage Ⅲa non-small cell lung cancer with N2 mediastinal node involvement. J Natl Compr Cancer Netw.

[8] Ripley RT, Rusch VW (2013). Role of induction therapy: surgical resection of non-small cell lung cancer after induction therapy. Thorac Surg Clin.

[9] Imai K, Matsuzaki I, Minamiya Y (2011). Postoperative bronchial stump fistula after lobectomy: response to occlusion with polyglycolic acid mesh and fibrin glue via bronchoscopy. Gen Thorac Cardiovasc Surg.

[10] Tayama K, Eriguchi N, Futamata Y (2003). Modified Dumon stent for the treatment of a bronchopleural fistula after pneumonectomy. Ann Thorac Surg.

[11] Li YD, Han XW, Li MH (2016). Bronchial stump fistula: treatment with covered, retrievable, expandable, hinged stents - preliminary clinical experience. Acta Radiol.

